The article "A Case of Acinetobacter junii Cavitary Pneumonia With Bacteremia in a Patient With Systemic Lupus Erythematosus" was published in 2021. Journal: Cureus.

# A Case of Acinetobacter junii Cavitary Pneumonia With Bacteremia in a Patient With Systemic Lupus Erythematosus

**DOI:** 10.7759/cureus.19711

**Published:** 2021-11-18

**Authors:** Sudarsan Kollimuttathuillam, Nyan Bethel, Hamid Shaaban

**Affiliations:** 1 Hematology and Medical Oncology, Saint Michael's Medical Center, Newark, USA; 2 Internal Medicine, Saint Michael's Medical Center, Newark, USA; 3 Hematology/Oncology, Saint Michael's Medical Center, Newark, USA

**Keywords:** bacteremia, pneumonia, lupus, sle, a. junii, acinetobacter

## Abstract

*Acinetobacter* genus includes multiple species, most notably *A. baumanii* that constitutes a common cause of nosocomial infections worldwide, particularly in patients with underlying immunodeficiency and risk factors (e.g., prior broad-spectrum antibiotic therapy, central venous catheter, mechanical ventilation). *A. junii* is a very rare human pathogen that is particularly associated with outbreaks of sepsis in immunocompromised neonates and pediatric oncology patients and rarely in immunocompromised adults. To our knowledge, this is the first case report of cavitary pneumonia with bacteremia secondary to *A. junii* in a patient with systemic lupus erythematosus (SLE).

## Introduction

*Acinetobacter junii* can cause serious infections, but they are generally non-fatal because the micro-organism is commonly susceptible to antimicrobial agents [1-3].

*Acinetobacter* species are aerobic gram-negative coccobacilli that have emerged as important opportunistic pathogens, especially among severely debilitated patients [2]. Earlier also known as *A. agrimoniin, A. junii* is a rare human pathogen, being particularly associated with outbreaks of septicemia in neonates and pediatric oncology patients [3-5]. The true incidence of infections by *A. junii* might be underestimated, since phenotypical identification is difficult and may require analysis of 16S rDNA or DNA-DNA-hybridization studies. To our knowledge, we are presenting the first rare case of *A.junii* pneumonia with bacteremia in a patient with systemic lupus erythematosus (SLE).

## Case presentation

A 47-year-old smoker with recently diagnosed SLE treated with intravenous cyclophosphamide and steroids who presented to the emergency department with complaints of a one-week history of non-productive cough associated with chills and a two-day history of right-sided pleuritic chest pain and shortness of breath.

He worked in a warehouse handling packages. On physical examination, the patient was in moderate respiratory distress; his blood pressure was 140/62, heart rate = 97, temperature = 96.8, RR = 35, O2 saturation = 92% on 4L nasal cannula. Skin examination revealed multiple skin tattoos. He had a papular malar rash and scaly plaques on the extensor aspects of both upper and lower limbs. His finger examination revealed clubbing. Chest examination revealed decreased air entry bilaterally, increased rhonchi and rales in the right upper lobe and left lower lobe areas. No pleural or pericardial rubs were appreciated.

The article "A Case of Acinetobacter junii Cavitary Pneumonia With Bacteremia in a Patient With Systemic Lupus Erythematosus" was published in 2021. Journal: Cureus.

During the first four hours, he developed severe respiratory distress and was intubated. Initial chest X-ray showed a left upper lobe consolidation. CT scan of the chest (Figure 1) demonstrated a 9 x 7 x 7 cm consolidation in the left upper lobe, with a honeycombed appearance. There was moderate paraseptal emphysema at the lung apices. The patient was admitted to the intensive care unit and blood and respiratory cultures were sent. He was initially started on vancomycin 1000 mg every 12 hours, meropenem 500 mg IV q 12 hours, and levofloxacin 750 mg Q48H for the treatment for healthcare-associated pneumonia (HCAP) in an immunocompromised patient. For the active SLE flare, he was given 500 mg IV methylprednisolone daily for three days, followed by steroid taper over two weeks. Emergent dialysis for severe metabolic acidosis secondary to rapidly progressive renal failure was begun. Additionally, tbo-Filgrastrim for neutropenia and intravenous immunoglobulin for thrombocytopenia were administered. The patient has also transfused three units of packed red blood cells and platelets. Initial blood and respiratory cultures grew gram-negative rods. Subsequently, DNA-DNA-hybridization studies were done and the organisms were identified as *Acinetobacter junii*. The organism was sensitive to all antibiotics tested except cefazolin. For the first 72 hours, the patient was treated with meropenem 1000 mg IV Q24H. When final results of the cultures were available, the regimen was changed to ciprofloxacin daily for two weeks.

**Figure 1:** CT of chest revealing left upper lobe cavitary pneumonia.

He responded well to antimicrobials and repeat blood cultures were negative. He had a prolonged ICU course during which he was ventilator dependent and received multiple sessions of dialysis for renal failure. He required a tracheostomy and had a tunneled dialysis catheter placed. The patient’s hospital course was stable till day 23 of hospitalization where he developed complications of SLE in the form of alveolar hemorrhage. The patient later developed multi-organ failure and died.

## Discussion

*Acinetobacter *species are opportunistic pathogens causing nosocomial infections [6]. Relatively few infections caused by *Acinetobacter* spp. are community-acquired, reported primarily from countries with tropical or subtropical climate, and mainly affected patients with some form of comorbidity or associated with heavy smoking and excess alcohol consumption [7]. Clinical forms of *Acinetobacter* infections include mainly the respiratory tract, blood-stream infections, peritoneum, urinary tract infection, surgical wounds, meningitis, skin and soft tissue infections and eye infections.

The article "A Case of Acinetobacter junii Cavitary Pneumonia With Bacteremia in a Patient With Systemic Lupus Erythematosus" was published in 2021. Journal: Cureus.

The majority of *Acinetobacter spp. *are* A. baumannii*, followed by *A. lwoffii. A. junii* accounts for less than 1% of isolates [8]. Although these infections are mainly attributed to *Acinetobacter baumannii *as a clinically and epidemiologically most important pathogen of the genus. Other *Acinetobacter spp.* are also being increasingly recovered from clinical specimens. *Acinetobacter* spp. raise alarm due to the extent of their antimicrobial resistance which may be exerted against almost all antibiotics currently in use, including the last-line antibiotics like cephalosporins, aminoglycosides, fluoroquinolones, and carbapenems. Notably, multi-resistant clinical *Acinetobacter *isolates other than *A. baumannii* are being increasingly reported worldwide. In addition to their biochemical properties, isolates are classified into different species based on sequencing of the 16S ribosomal ribonucleic acid (rRNA) gene.

*Acinetobacter junii *was first described in 1986 based on biochemical characteristics as a genomic species that were unable to oxidize glucose and able to utilize DL-lactate and L-histidine but not glutarate or azelate [9]. A few strains which were initially classified as *A.grimantii* were later reclassified as *A. junii* MTCC 11364 based on genomic sequencing [10].

Few reports on *A. junii* bacteraemia have been published. A few reports of nosocomial outbreaks caused by *A. junii* have been described. The first study described an outbreak in a neonatal ICU and IV fat emulsion was implicated as the possible source [11]. The second study described the outbreak in Paediatric Oncology ward and aerators were implicated as the source [12]. A single case report on *A. junii* bacteremia in an adult immunocompetent patient was also seen [13]. Corneal ulcer and perforation [14,15], peritonitis in peritoneal dialysis patients [16], meningitis [7] have also been described. Henao-Martinez et al. described a case of community-onset non-traumatic cellulitis caused by a strain identified as *A. junii-johnsonii* [17].

The largest study on *A.junii* bacteraemia is a case series of 43 patients in a period of 2000-2009 in Taiwan, most of the described patients had central venous catheters (80%) and almost all of them acquired infection during hospitalization [18]. More than half of cases of *A. junii* bacteremia were associated with impaired immunity (leukemia/lymphoma or solid tumors). Three patients in this study had AIDS/autoimmune disease-causing immunosuppression. A previous study evaluating the clinical characteristics of patients with *A. junii *infections also reported that this pathogen mainly affected patients who have had prior antimicrobial therapy, invasive procedures or malignancy [4]. There have been case reports of *A. junii* infection in adult oncology patients as well as post bone marrow transplantation [5,19]. In all studies, the infections primarily manifested as bacteremia in a majority of cases. Although *A. junii* is capable of causing serious infections, they are generally non-fatal because the micro-organism is commonly susceptible to antimicrobial agents. [11] Clinical presentation with septic shock within a week on *A. junii* infection has been described as an adverse prognostic factor.

The article "A Case of Acinetobacter junii Cavitary Pneumonia With Bacteremia in a Patient With Systemic Lupus Erythematosus" was published in 2021. Journal: Cureus.

Unlike *A. baumanii*, which is notorious for multidrug resistance, *A. junii* usually is sensitive to most antibiotics. In a case series, all isolates were susceptible to carbapenem and levofloxacin. More than 95% of the isolates were susceptible to amikacin and ciprofloxacin. Curiously in the same study, the authors noted that over the study period, a significant proportion of strains developed Colistin resistance (35%). Carbapenem-resistant* A. junii* infections have been recently reported in the literature [20]. 

Our patient had the perfect setting for *A. junii *infection. First, the patient had a hospitalization predisposing him to acquire the bacterial infection. We were not able to specifically identify the source. Secondly, he had an immunocompromised state in the setting of steroids, cyclophosphamide and an underlying autoimmune disorder. The strain isolated was susceptible to most antibiotics confirming with the previous studies. The patient never went into clinical shock and clinically improved within a few days of therapy with ciprofloxacin. However, this case is somewhat unique because of the clinical presentation of *A. junii* bacteremia and cavitary pneumonia in an SLE patient with no previous indwelling venous catheterization.

## Conclusions

This case highlights the importance of considering rare organisms such as *Acinetobacter junii* as a cause of multilobar cavitary pneumonia in immunocompromised patients because early identification by genomic studies may potentially lead to early treatment and intervention to improve outcomes.
